This article has been retracted.

# Using Plasma Autoantibodies of Central Nervous System Proteins to Distinguish Veterans with Gulf War Illness from Healthy and Symptomatic Controls

**DOI:** 10.3390/brainsci10090610

**Published:** 2020-09-05

**Authors:** Mohamed B. Abou-Donia, Elizabeth S. Lapadula, Maxine H. Krengel, Emily Quinn, Jessica LeClair, Joseph Massaro, Lisa A. Conboy, Efi Kokkotou, Maria Abreu, Nancy G. Klimas, Daniel D. Nguyen, Kimberly Sullivan

**Affiliations:** 1 Department of Pharmacology and Cancer Biology, Duke University Medical Center, Durham, NC 27710, USA; donia@duke.edu (M.B.A.-D.); elizabeth.lapadula@duke.edu (E.S.L.); 2 Department of Neurology, Boston University School of Medicine, Boston, MA 02118, USA; mhk@bu.edu; 3 Departments of Biostatistics and Environmental Health, Boston University School of Public Health, Boston, MA 02118, USA; eq@bu.edu (E.Q.); jleclai2@bu.edu (J.L.); jmm@bu.edu (J.M.); ddn@bu.edu (D.D.N.); 4 Department of Medicine, Harvard Medical School, Boston, MA 02115, USA; lisa_conboy@hms.harvard.edu (L.A.C.); ekokkoto@bidmc.harvard.edu (E.K.); 5 Dr. Kiran C. Patel College of Osteopathic Medicine, Institute for Neuroimmune Medicine, Nova Southeastern University, Fort Lauderdale, FL 33314, USA; mariamercedesabreu@gmail.com (M.A.); nklimas@nova.edu (N.G.K.); 6 Department of Immunology, Miami VA Medical Center, Miami, FL 33125, USA

**Keywords:** etiology, Gulf War Illness, CNS autoantibodies, myalgic encephalomyelitis/chronic fatigue syndrome, irritable bowel syndrome

## Abstract

For the past 30 years, there has been a lack of objective tools for diagnosing Gulf War Illness (GWI), which is largely characterized by central nervous system (CNS) symptoms emerging from 1991 Gulf War (GW) veterans. In a recent preliminary study, we reported the presence of autoantibodies against CNS proteins in the blood of veterans with GWI, suggesting a potential objective biomarker for the disorder. Now, we report the results of a larger, confirmatory study of these objective biomarkers in 171 veterans with GWI compared to 60 healthy GW veteran controls and 85 symptomatic civilian controls (*n* = 50 myalgic encephalomyelitis/chronic fatigue syndrome (ME/CFS) and *n* = 35 irritable bowel syndrome (IBS)). Specifically, we compared plasma markers of CNS autoantibodies for diagnostic characteristics of the four groups (GWI, GW controls, ME/CFS, IBS). For veterans with GWI, the results showed statistically increased levels of nine of the ten autoantibodies against neuronal “tubulin, neurofilament protein (NFP), Microtubule Associated Protein-2 (MAP-2), Microtubule Associated Protein-Tau (Tau), alpha synuclein (α-syn), calcium calmodulin kinase II (CaMKII)” and glial proteins “Glial Fibrillary Acidic Protein (GFAP), Myelin Associated Glycoprotein (MAG), Myelin Basic Protein (MBP), S100B” compared to healthy GW controls as well as civilians with ME/CFS and IBS. Next, we summed all of the means of the CNS autoantibodies for each group into a new index score called the Neurodegeneration Index (NDI). The NDI was calculated for each tested group and showed veterans with GWI had statistically significantly higher NDI values than all three control groups. The present study confirmed the utility of the use of plasma autoantibodies for CNS proteins to distinguish among veterans with GWI and other healthy and symptomatic control groups.

## 1. Introduction

Although the 1991 Gulf War (GW) only had less than two months of air strikes and less than a week of ground combat, approximately one-third of the 697,000 U.S. veterans developed a combination of health symptom complaints, including debilitating fatigue, chronic headache and body pain, memory and concentration difficulties, gastrointestinal problems, and skin abnormalities, known as Gulf War illness (GWI) [1,2,3]. In addition, some GW veterans also had increased rates of two other distinct conditions, Irritable Bowel Syndrome (IBS) and Myalgic Encephalomyelitis/Chronic Fatigue Syndrome (ME/CFS), which have overlapping symptoms with GWI [4,5]. Given these overlapping symptoms with other chronic conditions, it has been difficult to confirm the presence or absence of GWI or to differentiate between these disorders [6,7,8]. Neuroimaging has been found to be useful as a differential diagnostic tool for GW ill versus GW healthy individuals; however, what has been missing is the ability to use a less invasive, more readily available, and less costly tool, such as blood biomarkers to differentiate GWI from GW healthy status and differentiate GWI from another chronic multisymptom discord [6,8]. There have been some encouraging blood biomarker studies reporting differences between GWI cases and controls on neuroinflammatory markers that require validation in other GWI cohorts [9,10,11]. In addition, recently, we reported on a pilot study of serum biomarkers, which found seven out of eight markers significantly differed in veterans with GWI versus symptomatic controls with lower back pain, suggesting new potential blood markers for GWI [12]. The current study expanded on these prior findings by adding newly developed cutting-edge blood plasma autoantibodies in GW veteran and civilian cohorts, including those with IBS and ME/CFS, to identify whether veterans with GWI have the signature central nervous system (CNS) damage associated with their deployment that is different from other groups with overlapping chronic symptoms. IBS is a chronic mutisymptom illness that affects the gastrointestinal system and results in diarrhea or constipation or both. Although the cause of IBS is not known, it may result from altered gut motility, stress, environmental exposures, and genetic predisposition. It has also been shown to be related to alterations of the gut–brain axis in animal models of GWI and in a pilot study of GW veterans [13,14,15,16]. ME/CFS is characterized by extreme fatigue, muscle pain, headaches, multijoint and throat pain, lymph node swelling and soreness, chronic insomnia, and sleep disorders [6]. In addition, it may cause loss of memory and reduced concentration. Contributing factors may include viruses, weakened immune system, stress, or environmental exposures. Although some symptoms among the three disorders (GWI, IBS, ME/CFS) overlap, the etiologies differ, raising the question whether objective blood markers of GWI could be distinguished among these other chronic medical conditions.

GW veterans were exposed to numerous environmental neurotoxicants, including acetylcholinesterase (AChE)-inhibiting organophosphate pesticides and nerve gas agents [17,18]. Early studies investigated the hypothesis that GWI resulted from combined exposures of GW-relevant toxicants including pyridostigmine bromide (PB), *N*,*N*-diethyl-meta-toluamide (DEET), permethrin, and chlorpyrifos in hens [19,20]. Mixed exposures to multiple toxicants resulted in significantly greater toxic effects than separate exposures. More recent results with GW veterans who were pesticide applicators during the war also showed that combination exposures to PB and pesticides were associated with higher rates of GWI and specifically, with diminished CNS functioning on mood and cognition [18].

Pesticides used during the GW easily enter through the blood–brain barrier (BBB) because they are lipid-soluble [19,20]. These neurotoxicants have been found to be associated with autoantibodies to CNS proteins in the blood in several prior studies and exposed groups [12,20,21]. These exposures have been associated with neurological symptoms associated with CNS cellular functioning. For example, studies showed increased levels of CNS cellular proteins in pesticide-exposed participants with neurological symptoms [22,23,24]. These results were similar to those found in our pilot study of ill GW veterans [12].

The brain has two types of cells: neurons and supporting glial cells, including astrocytes and oligodendrocytes [21,25,26,27]. Neurons are characterized by the cell body and two additional parts, including axons and dendrites. Proteins in the axon include neurofilament triplet proteins (NFP), tubulin, tau, calcium/calmodulin kinase II (CaMKII), and (α-syn) [20,21,26,28]. Proteins in the dendrites include microtubule associate protein (MAP-2) [28]. Microtubules and tau make up the cytoskeleton of neurons.

Glial support cells include oligodendrocytes that myelinate axons using myelin basic protein (MBP) and myelin-associated glycoprotein (MAG). Astrocytes secrete glial fibrillary acidic protein (GFAP) and S100B only in the CNS [21,29,30].

The present study was carried out to use our newly developed biomarker test to differentiate GWI from other chronic conditions and healthy controls and confirm/validate our previous preliminary report of a small number of GW veterans and symptomatic controls showing increased CNS protein autoantibodies in their blood [12]. We hypothesized that as a result of neurotoxicant exposures during the war, autoantibodies to these ten CNS proteins would be increased in veterans with GWI when compared with other healthy and symptomatic control groups. Specifically, we hypothesized that neuronal and glial CNS proteins would differ in veterans with GWI compared with healthy and symptomatic controls with similar multisymptom disorders, including IBS and ME/CFS.

## 2. Materials and Methods

Study Population: GW illness consortium (GWIC) and the Dynamic Modeling of GWI study participants, two Department of Defense supported studies at Boston University and Nova Southeastern University, provided plasma samples from veterans deployed to the 1991 GW. Additional GWI participant samples were shared from the New England School of Acupuncture. These three established biorepositories of GW veterans were used from veterans who consented to share their blood samples for future studies. Control samples were provided by the Congressionally Directed Medical Research Program (CDMRP) funded studies in Boston and Florida, and samples from patients with Irritable Bowel Syndrome came from the biorepository at Beth Israel Deaconess Medical Center. Institutional Review Boards (IRBs) approvals from these biorepositories were obtained from Boston University, Nova Southeastern University, the Miami VA Medical Center, and Beth Israel Deaconess Medical Center.

The same standard operating procedures for phlebotomy, plasma separation, aliquoting, and storage were followed by all labs for all samples. Plasma samples were obtained from fasting subjects. Samples remained frozen at −80 °C until shipped for autoantibody analysis.

Cases and controls were determined by Kansas GWI criteria [31]. This criterion requires GW veterans to self-report symptoms in 3 out of 6 symptom domains (neurologic/mood/cognitive, fatigue, pain, gastrointestinal, respiratory, and skin). Veteran controls were deployed to the GW and did not meet the Kansas GWI or exclusionary criteria. Exclusions included CNS medical conditions and psychiatric illnesses that could account for their symptoms [31]. Plasma samples from symptomatic controls came from prior studies of individuals with ME/CFS and IBS. ME/CFS cases were determined by using 1994 CDC criteria [5]. IBS cases were determined by Rome III criteria [32]. The full cohorts have been described in previous papers (GWIC, ME/CFS, IBS, GWIC subsample) [4,12,14,33,34]. Institutional review boards at Nova Southeastern University/Miami VA Medical Center, New England School of Acupuncture, Beth Israel Deaconess Medical Center, and Boston University provided approval. All participants signed consent to use their plasma for follow-up studies of GWI biomarkers.

Ethical Statement: Approval for the use of stored blood samples for this study was obtained from the Duke University Health System Institutional Review Board for Clinical Investigations on 9 October 2017 and from the Boston University Medical Campus Institutional Review Board on 19 January 2018. The specific protocol components for Duke University were: Protocol ID: Pro00003202, Reference ID: 335940, Principal Investigator: Mohamed Abou Donia, Protocol Title: ‘Nervous System Injury’. The specific protocol components for Boston University were Protocol ID: H-34334, Reference ID: 1288716, Principal Investigator: Kimberly Sullivan, Protocol Title: ‘Novel Autoantibody Serum and Cerebrospinal Fluid Biomarkers in Veterans with Gulf War Illness’.

### 2.1. Materials

The proteins used in this study were as follows: Tubulin (human recombinant, Cat. #PRO-982, ProSpec-Tany TechnoGene Ltd., East Brunswick, NJ, USA), Microtubule-Associated Protein 2 (MAP-2, human recombinant, Cat. #TP316775, OriGene, Rockville, MD, USA), Tau-381 (human recombinant, Cat. #AG952, MilliporeSigma, Burlington, MA, USA), Neurofilament Protein (NFP, Cat #PRO-523, ProSpec-Tany TechnoGene Ltd., East Brunswick, NJ, USA), Calmodulin Kinase II (human recombinant, CaMKII, Cat #H000000H15-P01, Novus Biologicals, Littleton, CO, USA), Alpha-synuclein (human recombinant, Cat. #AS-55555, AnaSpec, Fremont, CA, USA), Myelin Basic Protein (MBP, human, Cat. #30R-AM030, Fitzgerald Industries International, Acton, MA, USA), Myelin-Associated Glycoprotein (MAG, human recombinant, Cat. #131–86-H02H, Sino Biological Inc., Wayne, PA, USA), Glial Fibrillary Acidic Protein (GFAP, human, Cat. #345996, CalBiochem, San Diego, CA, USA), and S100B Protein (human, Cat. #30R-AS002, MilliporeSigma, Burlington, MA, USA).

### 2.2. Procedures

Plasma procedures: All sites used the same written standard operating procedures for venipuncture, blood handling, plasma separation, aliquoting, and storage at −80 °C. Blood samples were collected prior to intervention for treatment trials. Samples remained frozen until sent for analyses and were visually inspected to not have hemolysis.

Western blot assay: In this study, a Western blot analysis was used for determination of CNS autoantibodies and antigens from the plasma samples of GWI cases and healthy and symptomatic controls. All plasma samples were analyzed three times for consistency and followed the protocol previously published in [12]. Specifically, each CNS protein was loaded into 10 ng/lanes. Immunoglobulin G (IgG) was loaded into a 100 ng/lane. All proteins were denatured and electrophoresed on SDS-PAGE (gradient 4% to 20% gradient) and a separate gel was used for each plasma sample. Enhanced chemiluminescence was used to determine if proteins were found by using a Typhoon 8600 variable model recorder (GE Lifesciences, Marlborough, MA, USA). The signal intensity was determined by Bio-Rad Quantity One image analysis software (Hercules, CA, USA). Specifically, the protein bands were quantified on digitized images in the mid-dynamic range using Quantity One software (Bio-Rad) and densitometry measurements were normalized to IgG in the same samples. Lab researchers were blinded to the case–control status of the samples.

### 2.3. Calculations

Measurement of chemiluminescent optical density for cases and controls was obtained by dividing plasma IgG concentrations. This optical density measure was normalized to controls and expressed as fold-change from healthy controls. Therefore, the CNS autoantibody measurements were presented as mean triplicate assay values normalized to healthy control values.

### 2.4. Neurodegeneration Index (NDI)

This new index was designed to determine the overall neurodegenerative condition of an individual based on the level of autoantibodies in the plasma. It is calculated by adding all of the values of autoantibodies for each neural protein, and then, dividing the sum by the number of autoantibodies used. Finally, this value is multiplied by 10 to produce the NDI.

Neurodegeneration Index (NDI) = (The Sum of Autoantibodies to “n” Proteins/n) × 10(1)

The NDI is used here as a simple, blood-based proxy to determine the extent of neurodegeneration of an individual, based on a plasma assay of autoantibodies for an individual.

### 2.5. Statistical Methodology

Descriptive statistics are presented as mean ± SE for continuous variables and as number and percent of participants per category of categorical variables. Subjects’ demographic values were compared across the four groups using one-way analysis of variance for continuous outcomes and the chi-square test for categorical outcomes. Mean values of the antibodies were compared across groups using analysis of covariance (ANCOVA) adjusting for age, sex, and race. *p* values were two-sided. To account for multiple comparisons, *p* < 0.001 was accepted as statistically significant for the comparisons between treatments on antibody levels. Analyses were conducted using SAS Version 9.4 (SAS Institute, Cary, NC, USA).

## 3. Results

### 3.1. Specificity of Serum Autoantibodies

The specificity of the serum autoantibodies against all tested neural proteins was previously reported by performing protein/peptide competitive assay [12,26]. The specificity of an autoantibody in the sera was assessed by performing a peptide/antigen absorption assay by preabsorbing the serum with the target proteins. The preabsorbed serum was tested by Western blot (Figure 1, Figure 2 and Figure 3).

### 3.2. Participant Demographics

Demographics are presented in Table 1. Participants were 175 veterans with GWI, 60 GW veteran healthy controls, 37 IBS controls, and 50 ME/CFS symptomatic controls. Significant differences were seen for age, sex, and race.

This study was carried out to use our newly developed neurodegenerative biomarkers to diagnose veterans of the 1991 Gulf War with GWI compared with healthy and symptomatic controls. The biomarkers consist of circulating autoantibodies of ten neural proteins (six neuronal and four glial) determined in the plasma of GW veterans with GWI, healthy Gulf war veterans, veterans with ME/CFS, and IBS that were used as controls. The NDI was calculated as described in the methods above and was assessed among the groups by chi-square tests.

### 3.3. Autoantibody Levels for Neuronal and Glial Proteins using Western Blot

Autoantibodies were determined for GWI cases, GW healthy veteran controls, IBS symptomatic controls, and ME/CFS symptomatic controls for the six neuronal proteins: NFP, tubulin, tau, MAP-2, CaMKII, and α-syn. In addition, four proteins from two types of glial cells were measured, including MBP and MAG from oligodendrocytes and GFAP and S100B from astrocytes.

The first analysis, which compared all three control groups combined (GW controls, IBS and ME/CFS groups), with veterans with GWI showed significantly increased mean levels for veterans GWI for nine out of the ten autoantibodies (Table 2; Figure 4). The only exception was for the glial protein S100B, whose mean level was similar to that of healthy controls (Table 2). In addition, there were no interacting the groups for any of the outcome measures.

The next analysis compared only GWI cases to GW veteran controls. The results of this comparison also showed that mean levels of nine out of the ten plasma autoantibodies of GWI cases were significantly higher for veterans with GWI than for healthy GW controls. Again, levels of S100B autoantibodies for GWI cases were not significantly increased from GW veteran controls.

Next, we compared GWI cases to symptomatic non-veteran IBS controls. The results again showed higher mean levels of nine out of ten autoantibodies for GWI cases compared to IBS controls. Again, the only non-significantly different autoantibody was S100B (Table 2).

Finally, we compared GWI cases to symptomatic non-veteran ME/CFS controls. The results showed higher mean levels of nine out of ten autoantibodies for GWI cases compared to ME/CFS controls. The only non-significantly different autoantibody between the two groups was for the GFAP protein (Table 2).

### 3.4. Neurodegeneration Index (NDI)

The Neurodegeneration Index score was calculated as described above for each tested group and the results were as follows (Figure 5): GWI = 39.35, GW healthy controls = 21.3, IBS controls = 11.94, and ME/CFS controls = 23.47. The mean NDI score for veterans with GWI was significantly higher than in all controls combined (*p* < 0.0001). In addition, the percentage of participants with NDI > 20 was significantly higher in GWI cases than in all controls combined (94.3% vs. 44.2%; *p* < 0.0001 via the chi-square test). The percentage of participants with NDI > 30 was also significantly higher in GWI cases than in all controls combined (71.8% vs. 14.3%; *p* < 0.0001 via the chi-square test).

## 4. Discussion

For the past 30 years, there has not been an objective diagnostic marker for GWI, which has hindered research in the field. Chronic symptoms reported by veterans with GWI have included headache, memory and attention decrements, debilitating fatigue, chronic pain, and gastrointestinal problems [2,3,35]. Many of these symptoms overlap with other comorbid conditions, including IBS and ME/CFS, necessitating the need for an objective marker that can delineate among these diagnostic groups. The present well-powered study confirms and expands the results of our previous descriptive study, where we identified a unique signature of objective biomarkers of CNS proteins in blood samples of 20 GW veterans compared with 10 controls [12]. In this study, we confirmed our prior results in a much larger sample of over 300 participants, including ill and healthy GW veterans and other symptomatic controls with IBS and ME/CFS. Specifically, we compared GWI cases vs. three control groups (GW controls, IBS, ME/CFS) and found that GWI cases had higher autoantibodies than all combined controls in nine out of ten autoantibodies. We then compared GWI cases with the three control groups separately and also found that the GWI cases showed significantly higher levels of nine out of ten autoantibodies than GW controls, IBS, or ME/CFS groups. These results clearly distinguish GWI cases not only from healthy GW counterparts but also other symptomatic controls with chronic multisymptom disorders.

Our results showed significantly elevated CNS autoantibodies in the plasma of veterans with GWI. The presence of low levels of autoantibodies in the plasma of GW healthy controls is consistent with previous findings in healthy individuals [12,36]. These results suggest that GW healthy controls had no lasting CNS effects from their deployment. In contrast, increased levels of CNS autoantibodies are consistent with veterans with GWI’s chronic neurological complaints and thus, provides an objective biomarker of the illness. The results revealed large increases in autoantibodies in the GWI cases compared to all controls except for S100B. These increases were significantly higher than controls with autoantibodies against MAP-2, showing the highest overall level in all groups tested. These were followed by autoantibodies against myelin and other glial-related proteins showing the highest levels (MAG > MBP > GFAP) and then, followed by increased neuronal cytoskeletal protein autoantibodies against Tubulin > NFP > Tau.

Our results show that autoantibodies to neural proteins can be used as biomarkers for diagnosis and prognosis of GWI and may also provide insight into the potential mechanisms of GWI. The only consistent risk factors for GWI are environmental exposures, including the use of pyridostigmine bromide pills and pesticides, which are now known to adversely affect the CNS in significant or combined dosages [14,15,17,18,19,20,24,25,26,27,28]. Although a total of over 50 pesticide products were used during the Gulf War, less than 20 were designated as “pesticides of concern” by the Department of Defense, including the insecticides permethrin and lindane as well as the repellant, DEET (*N*,*N*-diethyl-*m*-toluamide) and organophosphate insecticides and nerve gases, sarin and cyclosarin [23]. These same exposures were recently shown by our group to be associated with higher rates of GWI and specifically, with worse mood and cognitive functioning [18].

Furthermore, several studies have shown some organophosphorus (OP) compounds, such as sarin and chlorpyrifos in addition to inhibiting acetylcholinesterase, also cause neurodegeneration of the CNS [37,38,39,40]. A recent study reported increased CNS autoantibodies in blood from farm workers exposed to OP pesticides [41]. Investigations into the mechanisms by which these compounds cause neurodegeneration have established that OPs increase the activity and expression of CaMKII, which causes hyperphosphorylation of neural proteins, leading to their aggregation and slowing of axonal transport, resulting in neuronal cell death [19,42,43,44,45]. In agreement with this is our prior finding that airline crews who were exposed to OPs developed autoimmune antibodies to neural proteins [46]. Another study using Magnetic Resonance Imaging (MRI) examination of another cohort of aircrews, showed decreased white matter microstructure and blood perfusion are potential causes of cognitive and mood symptoms experienced by the aircrews [46].

These results suggest the involvement of white matter alterations in the development of GWI is consistent with increased autoantibodies against MBP and MAG that are present in myelinated axons [9,37,39,44]. Blood markers of MBP are also elevated in myelin-related CNS disorders. Increased autoantibodies to MBP in the plasma of veterans with GWI correlate with demyelination following axonal degeneration caused by exposure to OPs [12,37,39]. GFAP is a glial protein that is involved in white matter and blood–brain barrier functioning [21]. This finding also correlates with our recent finding that GFAP almost completely distinguished between GWI cases and controls in our prior pilot study [12]. This also correlates with recent findings of increased neuroinflammation seen in imaging the brains of veterans with GWI, as shown by significantly greater glial activation using PET brain imaging [47].

CaMKII is widely distributed in the CNS, constituting up to 2% of the protein in the hippocampus [48]. Exposure to organophosphates, such as di-isopropyl fluorophosphate (DFP), a surrogate compound for sarin, enhanced Ca^++^ release and increased expression and activity of CaMKII, resulting in hyperphosphorylation of several cytoskeletal proteins, i.e., tubulin, MAP-2, Tau, and neurofilament triplet proteins [44,45,49]. Increased phosphorylation of MAP-2, Tubulin, and Tau resulted in their aggregation and slowing of axonal transport [44,45,49]. CaMKII-induced hyperphosphorylation caused significant increase in both c-fos and c-jun expression, leading to apoptosis mediated by cytochrome c released from mitochondria due to the imbalance between the Bax, Bcl-2, and BCl-xl proteins triggered by the generation of Reactive Oxygen Species [29,30].

The results show that autoantibodies against S100B were not different from controls and were consistent with its neuroprotective action and the chronic nature of GWI. S100B’s half-life is 2 h in blood, supporting the use of its autoantibodies as biomarkers for neuronal conditions [29,30].

When the results of GWI cases were compared to controls with IBS, autoantibodies values were much higher, which is consistent with the fact that IBS is not considered a neurodegenerative disorder. The only elevated autoantibodies in IBS controls were against MAG but even that was less than half that of GWI cases. These results not only confirm the validity of our test as a biomarker for CNS effects, but also establishes its specificity as a marker for chronic GWI. MAG comes from oligodendrocytes in CNS and by Schwann cells in the periphery. The present results suggest that MAG protein was released from peripheral nerves in the gastrointestinal tract, a major target for IBS, suggesting its potential use for that disorder.

Furthermore, ME/CFS symptomatic controls exhibited levels of autoantibodies against neural proteins that were intermediate between veterans with GWI and controls with IBS. ME/CFS is characterized by body and muscle pains as well as some CNS symptoms, including debilitating fatigue. GWI cases had higher levels of all autoantibodies except for GFAP when compared with ME/CFS controls. The increased GFAP levels in ME/CFS suggest a potential marker and pathobiology for that disorder. Recent studies from other groups have shown increased antibodies against ß2-adrenergic receptors in ME/CFS patients [50,51]. This suggests that ME/CFS is more similar to GWI than IBS based on these autoantibody biomarkers, but GWI still clearly represents a unique disorder based on different autoantibody patterns.

Increased autoantibodies of biomarkers NFP, tau, tubulin, and MBP, and neuronal cytoskeletal disruptions, including microtubule instability, axonal degeneration, and altered axonal transport, have been found in many cell and animal studies of toxicant-induced models of GWI [27,42,43,44,45,49,52,53,54]. We are only aware of the following prior studies, including our prior pilot study, showing increased autoantibodies in much smaller pilot studies of GW veteran blood samples [12,55,56,57,58]. To our knowledge, this is the first large, more definitive study to validate these prior animal, cell, and veteran studies in the blood of ill GW veterans compared with combined and separate healthy and symptomatic comparison groups.

We hypothesized that exposures to chemicals present in the GW theater, such as pesticides and nerve gases, can cause CNS damage and release of CNS autoantibodies through the BBB into blood circulation, where B-lymphocytes produce antibodies to proteins and T cells produce cell-mediated immune responses, and IgG autoantibodies are then made [48,59,60]. Theoretically, IgG autoantibodies can enter through the BBB and disrupt CNS functioning, which could lead to symptoms of GWI [59,60,61]. Further research is needed to confirm this hypothesis. The results of the NDI analyses, showing GWI cases were three times more likely to have an NDI score of 30 or greater, suggest that these individuals may be at increased risk for early onset of age-related neurodegenerative disorders.

Correspondingly, recent studies have reported increased levels of CNS autoantibodies in blood, from neurodegenerative diseases such as Alzheimer’s disease (AD) and Parkinson’s disease (PD), suggesting the need for further studies of the potential increased risk of these disorders in GW veterans [62,63,64]. Having these reports, together with the results of the present study, raises concerns regarding the likelihood for veterans with GWI to develop neurodegenerative diseases such as AD and/or PD as they age. These CNS protein biomarkers may be useful for determining who is at risk for these disorders in addition to using them in clinical trials for treatment efficacy of GWI.

### Limitations

Like all studies, our study had limitations. GWI diagnosis was based on veterans’ self-reported symptoms, which could have introduced some classification errors. In addition, some veterans could have very early signs of neurodegenerative disorders that were not picked up in the clinical evaluations, which could have increased autoantibody levels in the veterans. However, the Kansas criteria for GWI would have excluded known cases of these disorders, including AD, PD, and other chronic illnesses that could have accounted for their chronic symptoms [31]. There were also sex differences within our groups as might be expected, with more women in the ME/CFS and IBS groups and more men in the GWI groups, and although these sex differences were controlled for in the analyses, future studies should more directly compare these autoantibody outcomes by sex. A major strength of our study included the large sample size and the inclusion of both healthy and symptomatic veteran groups in this objective biomarker study. In addition, the CNS autoantibody analyses were similar chronic multisymptom disorders (IBS, ME/CFS). We confirmed and validated our prior preliminary results of increased autoantibodies in a much larger sample of veterans with GWI compared with healthy GW veterans and with symptomatic non-veteran IBS and ME/CFS controls [12]. This study confirmed that nine of the ten autoantibodies were significantly increased in veterans with GWI, suggesting considerable CNS differences compared to both healthy and symptomatic controls. This confirms our prior studies, which suggested a strong CNS component to GWI [18,38]. The present study confirmed the utility of the use of plasma autoantibodies for CNS proteins to distinguish among veterans with GWI and other healthy and symptomatic control groups and our newly developed NDI summary score can be further utilized to compare pre and post treatment trial efficacy.

## Figures and Tables

**Figure 1:** Representative panel of Western blotting from three cases of the GWI patients (upper panels), and healthy controls (lower panels).

**Figure 2:** Representative panel of Western blotting from three cases of the IBS patients (upper panels), and healthy controls (lower panels).

**Figure 3:** Representative panel of Western blotting from three cases of the ME/CFS patients (upper panels), and healthy controls (lower panels).

**Figure 4:** Neural autoantibodies in plasma of GWI cases, GW healthy controls, IBS controls, and ME/CFS controls. *** *p* < 0.0001 (blue) GWI group to all three control groups combined using ANCOVA adjusted for age, sex, and race. *** *p* < 0.0001 (orange) GWI group to GW veteran control group using ANCOVA adjusting for age, sex, and race. *** *p* < 0.0001 (grey) GWI group to IBS group using ANCOVA adjusting for age, sex, and race. *** *p* < 0.0001 (yellow) GWI group to ME/CFS group using ANCOVA adjusting for age, sex, and race.

**Figure 5:** Neurodegenerative index score for GWI cases, GW healthy controls, IBS controls, and ME/CFS controls. Error bars represent the standard error of the mean. The mean NDI for GWI participants is significantly higher than in all controls combined (*p* < 0.0001).

**Table 1:** Demographic information of Gulf War Illness cases and healthy Gulf War and symptomatic controls.

Data	GWI Cases	GW Healthy Controls	IBS Controls	ME/CFS Controls
N	175	60	37	50
Age * (Mean ± SD)	48.7 ± 7.8	50.92 ± 7.48	39.40 ± 13.93	46.74 ± 10.24
Sex *				
Male (%)	80.2%	93.3%	8.6%	10%
Female (%)	19.8%	6.7%	91.4%	90%
Race *				
Caucasian (%)	81.3%	73.7%	85.7%	91.3%
African American (%)	12.9%	23%	8.6%	8.7%
Other/Multiracial (%)	5.8%	3.3%	5.7%	0.0%

Note: * denotes significant differences *p* < 0.01 across the four groups. We obtained information for age, sex, and race from 171 individuals for GWI veterans, and 35 individuals for IBS controls.

**Table 2:** Autoantibodies against neural proteins in GWI cases and healthy and symptomatic controls ^a^ using ANCOVA analysis and adjusting for age, sex, and race.

		GWI vs. All Controls	GWI vs. GW Controls	GWI vs. IBS Controls	GWI vs. ME/CFS Controls
A. Neuronal Proteins					
Neurofilament Triplet	Mean (SE)	3.42 (0.19) ***	1.88 (0.26) ***	0.86 (0.02) ***	1.18 (0.05) ***
Proteins (NFP)	Range	2.6–15.15	0.16–9.74	0.64–1.23	0.51–2.25
Tubulin	Mean (SE)	4.13 (0.25) ***	2.36 (0.30) ***	1.14 (0.03) ***	2.71 (0.24) **
	Range	0.32–15.15	0.09–10.76	0.62–15.36	0.63–7.39
Microtubule Associated Protein Tau (Tau)	Mean (SE)	2.92 (0.22) ***	1.57 (0.17) ***	1.24 (0.13) ***	1.02 (0.07) ***
	Range	0.33–10.55	0.34–5.13	0.52–4.11	0.40–3.36
Microtubule Associated Protein-2 (MAP-2)	Mean (SE)	9.66 (0.73) ***	5.04 (0.76) ***	1.05 (0.07) ***	6.97 (0.35) **
	Range	0.88–27.42	0.24–23.00	0.64–2.45	1.40–14.02
Calcium/Calmodulin	Mean (SE)	2.04 (0.15) ***	1.20 (0.13) ***	0.70 (0.03) ***	1.16 (0.05) ***
Kinase 2 (CaMKII)	Range	0.10–5.50	0.15–4.50	0.37–1.43	1.11–1.92
Alpha Synuclein (α-syn)	Mean (SE)	2.52 (0.19) ***	1.46 (0.02) ***	0.78 (0.06) ***	1.13 (0.05) ***
	Range	0.17–11.77	0.37–6.45	0.51–1.93	0.41–1.93
B. Glial Proteins: Oligodendrocytes					
Myelin Basic Protein (MBP)	Mean (SE)	4.28 (0.18) ***	2.17 (0.32) ***	1.19 (0.03) ***	1.52 (0.09) ***
	Range	0.09–17.34	0.42–11.83	0.74–1.7	0.44–4.33
Myelin Associated Glycoprotein (MAG)	Mean (SE)	4.94 (0.28) ***	2.12 (0.25) ***	3.20 (0.21) *	1.58 (0.11) ***
	Range	0.24–20.94	0.38–6.51	1.03–6.51	0.26–4/48
Glial Proteins: Astrocytes					
Glial Fibrillary Associated Protein (GFAP)	Mean (SE)	4.27 (0.18) ***	2.34 (0.30) ***	0.84 (0.03) ***	4.86 (0.26)
	Range	0.39–13.14	0.35–14.98	0.45–1.38	0.66–8.44
Glial S100B (S100B)	Mean (SE)	1.17 (0.04)	1.16 (0.03)	0.95 (0.03)	1.34 (0.06) *
	Range	2.60–2.41	0.37–2.74	0.53–1.34	0.49–2.26

Note: * *p* < 0.01 ** *p* < 0.001 *** *p* < 0.0001. ^a^ Values reflect fold change relative to control.
